# miR-218 inhibits the migration and invasion of glioma U87 cells through the Slit2-Robo1 pathway

**DOI:** 10.3892/ol.2015.2904

**Published:** 2015-01-27

**Authors:** JIAN-JUN GU, GUANG-ZHONG GAO, SHI-MING ZHANG

**Affiliations:** 1 Department of Neurosurgery, Taizhou People’s Hospital, Taizhou, Jiangsu 225300, P.R. China; 2 Department of Neurosurgery, The First Affiliated Hospital of Soochow University, Suzhou, Jiangsu 215006, P.R. China

**Keywords:** miR-218, gliomas, invasiveness, Slit2, Robo1

## Abstract

Malignant gliomas are the most common primary brain tumors in adults and are associated with the highest mortality rate. Glioma invasion is one of the most notable causes of the poor prognosis of this cancer. Preventing the invasive behavior of malignant glioma cells by altering effector molecules can significantly improve the prognosis of a patient. microRNAs (miRNAs) are small noncoding RNAs, ~22 nucleotides in length, that are able to function as oncogenes or tumor suppressors in human cancer. In the present study, the expression level of miRNA 218 (miR-218) was found to be markedly downregulated in glioma cell lines and human primary glioma tissues. miR-218 upregulation was found to dramatically reduce the migratory speed and invasive ability of glioma cells. Furthermore, it was demonstrated that ectopic expression of miR-218 in glioma cells resulted in the downregulation of roundabout, axon guidance receptor, homolog 1 (Robo1), upregulation of Slit homolog 2 (Slit2) and the expression of associated proteins following Robo1 knockdown by small interfering RNA. In addition, it was demonstrated that miR-218 inactivated the Slit2-Robo1 pathway through downregulating Robo1 expression by directly targeting the 3′-untranslated region (3′-UTR) of Robo1. The present results indicate that miR-218 plays important roles in preventing the invasiveness of glioma cells, and reveals a novel mechanism of miRNA-mediated direct suppression of the Slit2-Robo1 pathway in glioma.

## Introduction

Human gliomas originate from neural mesenchymal cells and account for 4–50% of nervous system tumors (1). The 2007 World Health Organization (WHO) classification (2) classifies astrocytomas as well-differentiated low-grade diffuse astrocytoma (WHO grade I-II), anaplastic astrocytoma (WHO grade III) and glioblastoma multiforme (GBM; WHO grade IV). Despite the use of aggressive surgery combined with radiation, chemotherapy and biological therapy (3), glioma remains a notable therapeutic challenge. There is an acknowledged requirement for novel therapeutic approaches based on an increased understanding of the biological and molecular nature of glioma (4).

microRNAs (miRNAs) are a class of short, non-coding single-stranded RNA molecules that are 22–25 nucleotides in length. miRNAs negatively regulate gene expression through the post-transcriptional silencing of target messenger RNAs (mRNAs), which occurs due to complementary binding (5,6). An increasing quantity of evidence has indicated an important role for miRNAs in the development of various cancers, including gliomas, and miRNAs have been associated with tumor suppressor and oncogenic activities (7,8). Among these miRNAs, miRNA 218 (miR-218) has been demonstrated to be downregulated in human GBM specimens compared with the adjacent tumor-free brain tissue (9–12). Accumulated evidence has revealed that upregulation of miR-218 can inhibit tumor cell invasion and proliferation in glioma cells by altering the expression of multiple target genes (12–15).

Previous studies have found that miR-218 inhibited the invasion and metastasis of gastric cancer by targeting the roundabout, axon guidance receptor, homolog 1 (Robo1) receptor and suppressing nasopharyngeal cancer progression through the downregulation of survivin and the Slit homolog 2 (Slit2)-Robo1 pathway (16,17). In the present study we examined how miR-218 affects the migration and invasion of glioma cells and the mechanism for miRNA-mediated direct suppression of the Slit2-Robo1 pathway in gliomas.

## Materials and methods

### Clinical samples

Tumor specimens were obtained from patients who underwent positive debulking surgery in the Neurosurgery Department of the The First Affiliated Hospital of Soochow University (Suzhou, China) between 2011 and 2013. The diagnosed gliomas were reviewed by an experienced neuropathologist, using histological slides, according to the 2007 WHO classification. The present study comprised 20 grade I–II, 20 grade III and 20 grade IV glioma samples. In addition, 10 normal brain tissue samples were obtained from internal decompression of patients with cerebral injury. This study complied with the requirements of the ethics committee of The First Affiliated Hospital of Soochow University and informed consent was obtained from all participants.

### Cell lines and transfection

Primary normal human astrocytes (NHA) were purchased from Sciencell Research Laboratories (Carlsbad, CA, USA). The U251, U87, SNB19 and LN229 glioma cell lines were obtained from the Institute of Biochemistry and Cell Biology (Shanghai Institutes for Biological Sciences, Chinese Academy of Science, Shanghai, China). The cells were maintained in RPMI-l640 medium containing 10% FBS, 50 units/ml penicillin G, and 250 μg/ml streptomycin (all purchased from Invitrogen Life Technologies, Carlsbad, CA, USA) in a humidified atmosphere containing 5% CO_2_, at 37°C. Transfections with miR-218 were performed in serum-free medium 24 h subsequent to plating, using Lipofectamine 2000 (Invitrogen Life Technologies). After 6 h, the cells were placed in complete medium and maintained at 37°C in a 5% CO_2_ atmosphere.

### Small interfering (si)RNA and transfection assays

Robo1-specific siRNA (forward, 5′-GGAUGUAUUUGCAAC AAGATT-3′ and reverse, 5′-UCUUGUUGCAAAUACAUC CTT-3′) was chemically synthesized by Qiagen (Hilden, Germany). The U87 cells were transfected with siRNA (HiPerFect Transfection Reagent; Qiagen) according to the manufacturer’s instructions. Briefly, the original stock of the siRNA was suspended in the siRNA suspension buffer provided by the manufacturer and stored at −20°C until use. On the day of transfection, 1×10^5^ cells were seeded in six-well plates (Corning Inc., Corning, NY, USA) with a total volume of 1,000 μl per well. siRNA was then gently introduced into the cells by adding 4 μl Oligofectamine™ Transfection Reagent (Invitrogen Life Technologies) and 5 μl siRNA (20 nM) per well. Non-silencing siRNA (GE Dharmacon, Lafayette, CO, USA) (forward, 5′-UUCUCCGAACGUGUCACGUTT-3′ and reverse, 5′-ACGUGACACGUUCGGAGAATT-3′) was used to control any effects of the transfection reagent and siRNA. The in vitro assays described herein were performed 24 h after transfection.

### RNA extraction and reverse transcription-quantitative polymerase chain reaction (RT-qPCR)

Total RNA, including miRNA, was extracted from the cultured cells or fresh glioma cancer tissues using TRIzol reagent (Invitrogen Life Technologies), according to the manufacturer’s instructions. The expression level of miR-218 was quantified using an miRNA-specific TaqMan miRNA Assay kit (Applied Biosystems, Foster City, CA, USA). U6 small nuclear RNA was used as an internal control. The mRNA expression of Slit2 and Robo1 was analyzed by qPCR, using the SYBR-Green method. All protocols were performed according to the manufacturer’s instructions and the results were normalized to the expression of GAPDH. The primer sequences were as follows: Slit2 forward, 5′-ACCTCT TGGCCAATCCTTTT-3′ and reverse, 5′-GAAGTCCTGAAT GGCCACAT-3′; Robo1 forward, 5′-GCCACCAGCAAGGAT GTATT-3′ and reverse, 5′-CCTGTAACATGGGCTGGAGT-3′; and GAPDH forward, 5′-TCGGAGTCAACGGATTTGG-3′ and reverse, 5′-CATGGGTGGAATCATATTGGA-3′.

### Western blotting

The cells were lysed in 1% Nonidet P-40 lysis buffer for 48 h following exposure to LY294002 or vehicle treatment. The homogenates were clarified by centrifugation at 20,000 × g for 15 min, at 4°C, and the protein concentrations were determined with a bicinchoninic acid protein assay kit (Pierce Biotechnology, Inc., Rockford, IL, USA). SDS-PAGE was performed on 40 μg of protein from each sample, the gels were transferred to polyvinylidene fluoride membranes (Merck Millipore, Darmstadt, Germany) and incubated with primary polyclonal goat anti-human Slit2 and rabbit anti-human Robo1 antibodies (1:200 dilution; sc-26599 and sc-25672, respectively, Santa Cruz Biotechnology, Inc., Dallas, TX, USA) followed by incubation with horseradish peroxidase-conjugated monoclonal goat anti-rabbit and donkey anti-goat secondary antibodies (1:1,000 dilution; cat nos. sc-2004 and sc-2020, respectively; Zymed Life Technologies, Carlsbad, CA, USA). The membranes were stripped using 1X phosphate-buffered saline with Tween 20 buffer (Wuhan Boster Biological Technology, Ltd., Wuhan, China) and reprobed with a primary monoclonal mouse anti-rabbit antibody against GAPDH (1:1,000 dilution; Bioworld, Nanjing, China). The protein bands were quantitated by densitometry using the gel analysis software ImageJ (National Institutes of Health, Bethesda, MA, USA. The values were normalized to GAPDH expression.

### Transwell assay and scratch-wound assay

Cell invasion was determined using Transwell and scratch-wound assays. For the Transwell assay, the appropriate oligonucleotides were transfected into the cells according to the aforementioned protocol. Subsequent to incubation for 48 h, 3×10^4^ cells were transferred to the top of the Matrigel-coated invasion chambers (BD Biosciences, San Jose, CA, USA) in a serum-free Dulbecco’s modified Eagle’s medium (DMEM). DMEM containing 10% fetal bovine serum was added to the lower chamber. After 24 h, the non-invading cells were removed, and the invading cells were fixed using 95% ethanol, stained with 0.1% crystal violet and images were captured under a ×100 magnification. The tests were repeated in three independent experiments. For the scratch-wound assay, the appropriate oligonucleotides were transfected into the cells in six-well plates. The cell layers were then scratched using a 200 μl sterile pipette tip to form wound gaps. The wound location in the six-well plates was marked. Images of the cells were captured to record the wound width at 0 and 24 h, and the images were captured at the marked wound location to measure the migratory ability of the cells.

### Luciferase assay

The 3′-UTR sequence of Robo1 predicted to interact with miR-218 or a mutated sequence with the predicted target sites was synthesized and inserted into the *Xba*I and *Fse*I sites of a pGL3 control vector (Promega Corporation, Madison, WI, USA). These constructs were named pGL3-Robo1–3′-UTR and pGL3-Robo1–3′-UTR-mut, respectively. For the reporter assay, the U87 cells were plated onto 24-well plates and transfected with pGL3-Robo1–3′-UTR or pGL3-Robo1–3′-UTR-mut and P-miR-218 or P-miR-control vectors using the FuGENE HD transfection reagent (Promega Corporation). A *Renilla* luciferase vector pRL-SV50 (Promega Corporation) was cotransfected to normalize the differences in transfection efficiency. Subsequent to 48 h transfection, the cells were harvested and assayed using the Dual-Luciferase Reporter Assay System (Promega Corporation), according to the manufacturer’s instructions. Transfection was repeated in triplicate in three independent experiments.

### Target prediction and network analysis

Robo1 was identified as a notable novel target of miR-218 using the conventional prediction tool, TargetScan (www.targetscan.org; Whitehead Institute for Biomedical Research, Cambridge, MA, USA).

### Statistical analysis

Experimental data were presented as the mean ± standard deviation. All analyses were performed using a two-tailed Student’s *t*-test performed on SPSS software, version 12.0 (SPSS, Inc., Chicago, IL, USA). P<0.05 was considered to indicate a statistically significant difference.

## Results

### miR-218 is downregulated in glioma tissues

To analyze the expression levels of miR-218, a qPCR analysis of miR-218 expression was conducted in the U251, U87, SNB19 and LN229 glioma cell lines. The present results revealed that miR-218 is downregulated in all glioma cell lines compared with the NHA cells (P<0.05). In addition, when miR-218 expression was measured in 10 normal brain tissue and 60 glioma tissue samples, it was observed that the expression level of miR-218 was significantly decreased in the glioma tissues, particularly in grade III/IV glioma tissues, compared with the normal brain tissues (Fig. 1). This result demonstrates that miR-218 expression decreases markedly between normal brain tissue and low grade to GBM tissue. Overall, the present results indicate that miR-218 is downregulated in glioma cell lines and glioma tissues.

### Upregulation of miR-218 inhibited cell invasion in U87 cells

As invasiveness is one of the pathophysiological features of human malignant gliomas, the effects of miR-218 on the invasiveness and migration of glioma cells were checked by Transwell and scratch-wound assays. An *in vitro* Matrigel invasion assay revealed that the invasiveness of U87 cells transfected with the miR-218 mimic was suppressed compared with control and NC groups (Fig. 2A and B). The results of the *in vitro* wound healing assay revealed that miR-218 significantly attenuated the migration of U87 cells compared with control and NC groups (Fig. 2C and D). This finding indicates that the upregulation of miR-218 inhibits the invasive ability of glioma cells *in vitro*.

### Upregulation of miR-218 reduces Robo1 expression via the inactivation of Slit2-Robo1 signaling

Development of invasiveness by malignant glioma cells involves multiple genetic alterations in signaling pathways. Numerous studies have reported that the Slit2-Robo1 signaling channels can inhibit glioma invasion and migration. However, the specific roles of Slit2/Robo1 in cancer cell invasion have not yet been completely elucidated *in vivo*. The present study also observed, using qPCR and western blot analysis, that treatment with the miR-218 mimic for 24 h significantly upregulated the expression of Slit2, which was followed by a decrease in Robo1 (Fig. 3). These results indicate that miR-218 reduced the expression of Robo1 via the inactivation of Slit2-Robo1 signaling.

### Robo1 is a functional downstream target of miR-218

A luciferase reporter assay further confirmed the direct interaction between miR-218 and the 3′-UTR of Robo1 mRNA (Fig. 4). The luciferase activity for the wild-type 3′-UTR of Robo1 was significantly inhibited by co-transfection with miR-218 mimics compared with constructs containing mutated 3′-UTRs. The present study demonstrated that Robo1 is a direct target of miR-218.

### Robo1 siRNA can imitate the role of miR-218 in U87 glioma cells

To assess the role of Robo1 in the miR-218-dependent inhibition of cell migration and invasion, miR-218 inhibitor was transfected into U87 cells treated with Robo1 siRNA. As expected, Robo1 protein expression was significantly reduced by the specific Robo1 siRNA (Fig. 5). The enhanced invasive ability of miR-218 inhibitor-transfected U87 cells declined when Robo1 siRNA was co-transfected with the miR-218 inhibitor (Fig. 6). These results indicate that Robo1 is essential for miR-218-dependent cell migration and invasion.

## Discussion

Malignant gliomas are diffuse tumors that are extremely invasive and usually multifocal. Glioma possesses a dismal prognosis, with a median survival of ~16 months (18). The ability for single tumor cell infiltration, which involves the extension of tendrils of the tumor several centimeters away from the main tumor mass, is one of the major obstacles for the effective treatment of gliomas, as this infiltration results in incomplete surgical removal and contributes to the high frequency of tumor recurrence (19). Despite the increasing quantity of evidence that demonstrates the promotion of glioma cell infiltration into the brain parenchyma by various stimuli, the mechanisms underlying the dysregulation of cell motility during tumor invasion by the insidious glioma cells have yet to be elucidated (20). As a result, exploring novel treatment methods is an urgent clinical challenge for neuroscientists.

Previous studies have revealed that miR-218 expression is often downregulated in several human cancers, including gastric cancer, lung squamous cell carcinoma, malignant astrocytomas and medulloblastomas, which indicates that miR-218 may function as a tumor suppressor (21–23). Studies have identified that the ectopic expression of miR-218 contributes to the inhibition of proliferation, invasion and migration in glioma cells, as well as the induction of apoptosis by downregulating the gene that was directly targeted by miR-218 (12–15). Firstly, miR-218 inhibits the expression of the target gene inhibitor of nuclear factor κB (NF-κB) kinase β, and in a dose-dependent manner, inhibits the expression of NF-κB, whilst reducing the expression of matrix metalloproteinase (MMP) 9 and inhibiting the invasion and migration ability of glioma cells (12). Secondly, epidermal growth factor receptor-coamplified and overexpressed protein (ECOP) has been identified as a functional downstream target gene of miR-218 that can regulate NF-κB transcription activity and is associated with the apoptotic response. Overexpression of miR-218 can restrain the activity of NF-κB through ECOP, thus inducing glioma cell apoptosis and inhibiting the activity, proliferation and tumorigenicity of glioma cells (13). Thirdly, the expression of lymphoid enhancer-binding factor 1 (LEF1) and MMP-9 in the high grade glioma group is extremely high, while the expression in the low-grade glioma group is extremely low, and is negatively correlated with the expression of miR-218. Overexpression of miR-218 inhibits the Wnt/LEF1 signaling pathways that lead to a reduction in MMP-9 synthesis, inhibiting tumor invasion (14). Finally, the abnormal expression of miR-218 in glioma cells decreased, but there was an abnormal increase in cyclin-dependent kinase (CDK) 6 expression, with the expression level of the two being negatively correlated. Overexpression of miR-218 in the glioma cell lines can inhibit CDK6 expression and glioma cell proliferation and promote its apoptosis (15).

Tumor development is a complex multi-step process that includes malignant tumor invasion and metastasis (24). The development of invasiveness in malignant glioma cells involves several genetic alterations within signaling pathways. Numerous studies have reported that the Slit2/Robo1 signaling channels can inhibit glioma invasion and migration. An *in vitro* study performed by Mertsch *et al* (25) identified, using a modified Boyden chamber assay, that the Slit2/Robo1 system serves as a chemorepellent for glioma cells, indicating that glioblastoma cells migrate away from increased Slit2 concentrations and prompt Robo1-positive glioma cell invasion along gray matter tracts and into white matter, including the corpus callosum (25). A previous *in vivo* study revealed that ectopic expression of Slit2 in SNB19 cells attenuates cell migration and invasion (20). These results indicate that Slit2/Robo1 can inhibit glioma invasion and migration *in vivo* and *in vitro*. Slit2 may also be a tumor suppressor gene that inhibits the migration and invasion of tumor cells and this inhibition appears to be mediated by Robo1 (20). Previous studies identified that miR-218 inhibited invasion and metastasis of gastric cancer by targeting the Robo1 receptor and suppressed nasopharyngeal cancer progression through the downregulation of survivin and the Slit2-Robo1 pathway (16,17).

In the present study, Robo1 was identified as a notable novel target of miR-218 using the conventional prediction tool TargetScan (www.targetscan.org). The expression levels of miR-218, Robo1 and Slit2 were detected in 70 tissue samples, consisting of normal brain tissue and low- and high-grade glioma tissues, using RT-qPCR and western blot analysis. It was found that the expression of miR-218 and Slit2 was always inverse to that of Robo1. Notably, the mRNA and protein levels of Robo1 were significantly decreased and the mRNA and protein levels of Slit2 were significantly increased subsequent to the transfection of miR-218 mimics into U87 cells. Furthermore, it was found that miR-218 was involved in modulation of the Slit2-Robo1 signaling pathway and downregulation of Robo1 expression by directly targeting the Robo1 3′-UTR. In addition, Robo1 siRNA can reduce the invasive ability of the cells subsequent to its enhancement by the exogenous expression of the miR-218 inhibitor. Overall, the present results indicate that miR-218 inhibits the migration and invasion of glioma cells through the Slit2-Robo1 signaling pathway. Therefore, the development miR-218 as a biomarker for glioma or as a potential therapeutic candidate for miRNA replacement therapy is extremely promising (26,27).

## Figures and Tables

**Figure 1:** miR-218 expression in glioma cells and tissues. (A) miR-218 expression was detected in the glioma U251, U87, SNB19 and LN229 and primary NHA cell lines. qPCR demonstrated that miR-218 was downregulated in all of the glioma cell lines compared with the NHA cells. ^*^P<0.05 vs. NHA cells. (B) miR-218 was detected in 10 normal brain and 60 glioma tissues by qPCR. miR-218 expression was significantly lower in glioma tissues compared with normal brain tissue. ^*^P<0.05 vs. normal brain tissue. miR-218, microRNA 218; NHA, normal human astrocytes; WHO, World Health Organization; qPCR, quantitative polymerase chain reaction.

**Figure 2:** miR-218 suppresses U87 cell invasion. (A and B) U87 cells were examined for cell invasion in 24-well plates with Transwell chambers. The migrated cells were stained with crystal violet. The invasiveness of U87 cells was attenuated with the upregulation of miR-218. (C and D) Images of the scratch-wound healing assay were captured at 0 and 24 h, and the wound gaps were analyzed by measuring the distance of migrating cells for three regions of each wound. ^*^P<0. 05. NC, negative control; miR-218, microRNA 218.

**Figure 3:** Upregulation of miR-218 reduces Robo1 expression through the inactivation of Slit2-Robo1 signaling. (A and B) The U87 cells were treated with control, NC and miR-218 mimics, and the levels of Robo1 and Slit2 mRNA were measured by quantitative polymerase chain reaction.(C) The level of Robo1 and Slit2 protein expression in the U87 cells was measured by western blot analysis. ^*^P<0. 05. Robo 1, roundabout, axon guidance receptor, homolog 1; Slit2, Slit homolog 2; NC, negative control; miR-218, microRNA 218.

**Figure 4:** Robo1 is a direct target of miR-218. (A) Identification of target sites in the 3′-UTR of Robo1 was performed using TargetScan. (B) A luciferase assay was performed to determine the target association in U87 cells transfected with the control pGL-3 vector, a vector containing the Robo1 sequence that was predicted to interact with miR-218 (Robo1-UTR) or a vector containing a mutated Robo1 sequence with the predicted target sites (Mu-Robo1-UTR). The reported data are representative of at least three independent experiments. ^*^P<0.05. Robo 1, roundabout, axon guidance receptor, homolog 1; UTR, untranslated region; miR-218, microRNA 218; NC, negative control.

**Figure 5:** Western blot analysis revealed that the protein expression of Robo1 was significantly increased in miR-218 inhibitor-transfected U87 glioma cells. By contrast, Robo1 siRNA decreased the miR-218 inhibitor-induced increase in Robo1 protein levels. ^*^P<0.05. Robo 1, roundabout, axon guidance receptor, homolog 1; NC, negative control; siRNA, small interfering RNA; miR-218, micro RNA 218.

**Figure 6:** In the U87 cell line, Robo1 siRNA reduced miR-218 inhibitor-induced enhanced invasive ability. (A and B) Transwell assays revealed that the miR-218 inhibitor promoted the invasion of U87 cells and Robo1 siRNA attenuated the invasion. ^*^P<0.05. (C and D) Robo1 siRNA attenuation of the migration of U87 cells was also observed in the scratch-wound assay. ^*^P<0.05. NC, negative control; siRNA, small interfering RNA; Robo1, roundabout, axon guidance receptor, homolog 1; miR-218, microRNA 218.
